RETRACTED

# Microbiome-Metabolomics Reveals Endogenous Alterations of Energy Metabolism by the Dushen Tang to Attenuate D-Galactose-Induced Memory Impairment in Rats

**DOI:** 10.1155/2021/6649085

**Published:** 2021-05-27

**Authors:** Jifeng Wang, Min He, Wenjun Guo, Yanhong Zhang, Xin Sui, Jianan Lin, Xiaoran Liu, Hui Li, Jing Li, Qing Yang, Mo Kan, Zhuang Zhang, Sitong Ming, Xiaobo Qu, Na Li

**Affiliations:** ^1^Jilin Provincial Key Laboratory of Biomacromolecules of Chinese Medicine, Jilin Ginseng Academy, Changchun University of Chinese Medicine, Changchun, Jilin 130021, China; ^2^Leiden University—European Center for Chinese Medicine, Leiden University, 2333CC Leiden, Netherlands; ^3^Qian Wei Hospital of Jilin Province, Changchun, Jilin 130117, China

## Abstract

Aging affects the brain function in elderly individuals, and Dushen Tang (DST) is widely used for the treatment of senile diseases. In this study, the protective effect of DST against memory impairment was evaluated through the Morris water maze (MWM) test and transmission electron microscopy (TEM). A joint analysis was also performed using LC-MS metabolomics and the microbiome. The MWM test showed that DST could significantly improve the spatial memory and learning abilities of rats with memory impairment, and the TEM analysis showed that DST could reduce neuronal damage in the hippocampus of rats with memory impairment. Ten potential biomarkers involving pyruvate metabolism, the synthesis and degradation of ketone bodies, and other metabolic pathways were identified by the metabolomic analysis, and it was found that 3-hydroxybutyric acid and lactic acid were involved in the activation of cAMP signaling pathways. The 16S rDNA sequencing results showed that DST could regulate the structure of the gut microbiota in rats with memory impairment, and these effects were manifested as changes in energy metabolism. These findings suggest that DST exerts a good therapeutic effect on rats with memory impairment and that this effect might be mainly achieved by improving energy metabolism. These findings might lead to the potential development of DST as a drug for the treatment of rats with memory impairment.

## 1. Introduction

Aging is one of the most important factors involved in the gradual functional decline and structural degeneration of the brain and has been implicated in memory impairment, which is a major symptom of Alzheimer's disease (AD) [1–3]. Due to the rapid aging of the population, memory impairment seriously affects the quality of life of a large number of elderly individuals [4, 5]. Recent studies of cerebral energy metabolism have shown that mitochondrial dysfunction, oxidative stress, excessive levels of advanced glycation end products, and neurotoxicity are involved in the pathogenesis of memory impairment [6, 7]. Studies of memory impairment and relevant pathogenesis mechanisms could provide novel perspectives and targets for exploring new drug candidates and new therapy strategies and for evaluating the efficacy of drugs against aging and AD.

RETRACTED

Traditional Chinese herbal medicines have shown unique therapeutic effects on various diseases. In China, Dushen Tang (DST, also called “Ginseng decoction”), which is composed of a single herbal material (Panax ginseng C.A. Meyer, regarded as “the king of herbs” in China), was first published in “Shi Yao Quan Shu,” which describes that its extraction method is decoction [8, 9]. DST has a long history of application and has been widely used, particularly for memory enhancement [10]. Modern pharmacological studies have confirmed the multiple pharmacological effects of ginseng, and these effects include memory enhancement, immune modulation, antioxidant stress, and antiaging effects [11]. Specifically, ginseng restores D-gal-induced memory deficits by enhancing hippocampal LPA1 receptor expression, LTP, and neurogenesis [12]. Ginseng polysaccharides and ginsenosides, which are the main active ingredients of the DST prescription, exert favorable curative effects on AD and other aging-related diseases [13–15]. However, the human body is a complicated system that exhibits dynamic metabolic changes and is affected by interactions between the intestinal flora and the host. Although the therapeutic effect of ginseng against memory impairments has been confirmed in clinical settings in China, the potential mechanism through which DST affects endogenous metabolism and the microbiome remains unclear.

Long-term injections of D-galactose (D-gal) have been widely used to establish AD and aging models because these cause many aging- or AD-like pathological symptoms, such as memory impairments, reduced neurogenesis, increased levels of amyloid precursor protein, and oxidative damage [1, 16, 17]. Using such an animal model might aid the assessment of therapeutic effects and could provide more scientific evidence and biological interpretations of the effects of DST against memory impairment.

Metabolomics analyzes the small molecules in a biological sample, such as serum and urine, to elucidate associations between metabolites and research subjects and elucidate the aberrant metabolic pathways involved in complex diseases, and as a result, this approach can efficiently screen biomarkers and allow an in-depth analysis of the molecular mechanisms regulating health or disease [18]. However, host metabolism is regulated not only by its own genome but also by its symbiotic bacteria, and among these bacteria, the gut microbiota both participate in and regulate metabolic processes [19]. The combination of metabolomics and microbiological techniques could provide a powerful tool to further study the relationship between host metabolism and the gut microbiota and to unravel the metabolic phenotype variations associated with the gut microbiota perturbations in disease development [20].

RETRACTED

A recent study illustrated the essential roles of the gut microbiota in central nervous system diseases, including Parkinson's disease, autism spectrum disorders, and AD [21]. A novel strategy of integrating 16S rRNA gene sequencing with UPLC-MS-based metabolomics has been applied to analyze the relationship among the gut microbiota, metabolites, and memory impairment [22–24], but this strategy has not been used to study the protective effects of DST against memory impairment induced by D-galactose in rats. Therefore, in this study, we used a rat model with memory impairment induced by D-galactose to study the potential protective effects of DST. These effects were assessed by the MWM test and transmission electron microscopy (TEM). Thereafter, the serum metabolites and the fecal microbial community were analyzed by UPLC-Q-TOF/MS and 16S rDNA, respectively. Multivariate statistical analyses, such as PLS-DA and principal coordinates analysis (PCoA), were used to identify specific biomarkers and to explore the changes in the gut microbiota, and the metabolic pathways related to memory impairment were explored using the KEGG database. An analysis combining the common changes in the flora and metabolites showed that DST can influence memory impairments by regulating several important intestinal bacteria and endogenous energy-related metabolites.

## 2. Materials and Methods

### 2.1. Materials and Preparation of Water Extracts of DST

Free-growing ginseng (natural dry rhizome of Panax ginseng C.A. Mey grown in a forest for 15 years) was purchased from Jilin zhi 'en tang ginseng special products Co., Ltd. China, and was validated by Dacheng Jiang (affiliated with the Changchun University of Chinese Medicine). The purchased ginseng (50 g) was immersed in 500 mL of deionized water for 2 h and then decocted three times (100°C, each extraction was conducted for 1 h). The decoction was filtered, combined together, and then condensed to 200 mL to obtain the final water extract.

### 2.2. Identification of the Main Compounds of DST

DST was transferred into a centrifuge tube and lyophilized with a freeze dryer. One hundred milligrams of the retained pellet was dissolved in 10 mL of 70% methanol solution and centrifuged at 14000 × g and 4°C for 10 min. A 4 *μ*L of aliquot of the supernatant was used for LC-MS analysis. Five milligrams of ginsenosides R1, Rg1, Re, Rf, Rh1, Rb1, Rc, Ro, Rb2, and Rb3 was weighed and placed in a 100 mL of volumetric flask. Methanol was added, and the volume was increased to the mark on the tube to obtain the reference solution. A 4 *μ*L of aliquot of the reference solution was used for LC-MS analysis.

RETRACTED

Chromatographic separation was performed using a Vanquish Duo UHPLC system (Thermo Fisher Scientific, San Jose, CA, USA) with a Hypersil GOLDTM column (2.1 mm × 50 mm, 1.9 *μ*m) at 30°C and an injection volume of 4 *μ*L. The mobile phase consisted of 0.1% aqueous formic acid (phase A) and acetonitrile (phase B) and was administered using the following gradient program with a flow rate of 0.4 mL/min: 10% B (0-4 min), 10-25% B (4-8 min), 25-29% B (8-16 min), 29% B (16-25 min), 29-95% (B 25-27 min), and 95% B (27-30 min).

Mass acquisition was conducted with a Q-Orbitrap mass spectrometer equipped with an electrospray ionization (ESI) source (Thermo Fisher Scientific, San Jose, CA, USA) operating separately in the negative ion mode, and the profile data were recorded in the range of m/z 200-1500. Full-scan acquisition was performed at a resolution of 7000, whereas tandem MS information was acquired under the ddMS2 mode with a resolution of 35000. The key parameters of the ionization source were set as follows: capillary voltage, -3.5 kV in the negative ion mode; sheath gas flow, 60 arb; auxiliary gas flow, 15 arb; sweep gas flow, 2 arb; and capillary temperature, 320°C. Prior to sample analysis, the mass spectrometer was calibrated using the vendor-provided Pierce™ calibration solution (Thermo Fisher Scientific, San Jose, CA, USA). All samples were maintained at 4°C through the analysis.

The LC-MS raw chromatographic data were processed using the TraceFinderTM (TF) software from Thermo Fisher Scientific. The main compounds of DST were identified by matching the obtained data with accurate mass and MS/MS information of natural products acquired from Orbitrap Traditional Chinese Medicine Library (OTCML) databases, and some of these compounds were identified using reference substances.

### 2.3. Animal Modeling and Treatments

A total of 30 healthy adult male Sprague-Dawley rats (six weeks old, weighing 200 ± 10 g) were purchased from Changchun Yisi Experimental Animal Technology Co., Ltd. (China, License No.: SCXK(Ji)-2018-0007). After one week of adaptation feeding, the rats were randomly divided into the following three groups (10 rats in each group): healthy control group, model group, and DST group. All the rats had free access to standard rodent chow and water. The model and DST-treated rats were intraperitoneally injected with D-gal (daily dose of 500 mg/kg) for 7 weeks. Additionally, the rats in the DST group were orally administered DST (0.3 g/kg/d) during the experimental period, and the rats in the control and model groups were administered the same volume of saline.

RETRACTED

### 2.4. Morris Water Maze Test

The MWM test was utilized to evaluate the spatial learning and memory capacities of the rats. This test forces rats to swim in water until they find a platform hidden underwater. Before the formal experiment, a training trial was conducted once per day for one week. On the test day, the rats were maintained on the platform for 10 s and then released in any of the four quadrants (once in each quadrant). The timer was set to 120 s, and the escape latency was time when the rat found the platform (up to 120 s). All behavioral data were obtained and examined using the SMART V3.0 video tracking system (Panlab Harvard Apparatus, Hugstetten, Germany).

### 2.5. Detection of Ultrastructural Changes in the Rat Hippocampus by Transmission Electron Microscopy

After the MWM test, the rats were perfused successively with 0.9% saline, 4% paraformaldehyde, and 1% glutaraldehyde via the heart. The skull was exposed, and the hippocampus was stripped, fixed in 2% paraformaldehyde-2.5% glutaraldehyde solution for 3 h at 4°C, washed thoroughly with 0.1 mol/L PBS, and fixed with 1% osmium tetroxide at 4°C for 1.5 h. After dehydration and embedding, semiultrathin sections with a thickness of 1-2 *μ*m were prepared. The hippocampus was stained with methylene blue and positioned under an optical microscope, and ultrathin sections of 50–70 nm were prepared. After staining with uranyl acetate and lead citrate, the ultrastructure of hippocampal neurons was observed under a transmission electron microscope.

### 2.6. Metabolomic Analysis

Serum samples (100 *μ*L) were extracted using methanol/acetonitrile/water (2 : 2 : 1, v/v), vortexed and shaken for 5 min, and centrifuged at 13,000 × g and 4°C for 15 min, and 100 *μ*L of aliquots of the supernatant was obtained, freeze-dried, mixed well with 100 *μ*L of water, and used for LC-MS analysis. Quality control (QC) samples were prepared by pooling equal volumes (10 *μ*L) of serum from each sample for optimization of the chromatographic and MS conditions. Subsequently, a 10 *μ*L of serum sample was analyzed using an Agilent 1290 Ultra Performance LC system equipped with a HILIC C18 column (Waters, ACQUITY UPLC BEH 100 mm × 2.1 mm, 1.7 *μ*m) at 25°C. Phase A was aqueous and consisted of 25 mM of ammonium acetate, and phase B was acetonitrile. The mobile phase was administered using the following gradient program at a flow rate of 0.3 mL/min: 95% B (0–0.5 min), 95%–65% B (0.5–7 min), 65%–40% B (7–9 min), 40% B (9–10 min), 40%–95% B (10–11.1 min), and 95% B (11–16 min). All the samples were maintained at 4°C until further analysis.

RETRACTED

Under the positive and negative ion modes, data were acquired over a full scan (range: 60–1200 Da) and MS2 scan (range: 25–1200 Da) using a Triple-TOF 5600 (AB SCIEX, USA) mass spectrometer. The mass spectrometry conditions consisted of the following: electrospray ionization (ESI); capillary voltage, 5.5 kV (ESI±); ion source gas 1, 60; ion source gas 2, 60; curtain gas, 30; and source temperature, 600°C.

The processed dataset was then fed to the SIMCA-P software package (v13.0, Umetrics, Umea, Sweden), and the normalized data were then used for principal component analysis (PCA) and partial least squares-discriminate analysis (PLS-DA). A PCA of the QC data was performed to evaluate the stability of the instrument, and PLS-DA was employed to characterize the metabolic perturbations among different groups. The features were filtered based on the variable importance in projection (VIP) values (VIP > 2) and fold change values (FC > 2) obtained from the initial group comparisons. Student's *t*-test was further applied to assess the significances of the differences in these features between groups using the GraphPad Prism 6.0 software (La Jolla, CA, USA). A value of *p* < 0.05 was considered to indicate statistical significance, and this criterion was used for the selection of biomarkers. The MetaboAnalyst software, which is a web-based tool for the visualization of metabolomic data, was used for the metabolic pathway analysis, and Impala network tools were used to predict signal pathways.

### 2.7. Microbial Community Analysis

Rat feces were collected and immediately stored at -80°C. Prior to DNA extraction, the samples were thawed and mixed well. Microbial DNA was extracted using the E.Z.N.A. to analyze the taxonomic composition of the bacterial community. An aliquot (200 mg) of each fecal sample was suspended in a mixture of 40 *μ*L of 10% N-lauroylsarcosine, 0.1 M Tris (pH 7.5), and 250 *μ*L of guanidine thiocyanate. The universal primers 338F and 806R were used to amplify the 16S rDNA gene using a PCR machine. For library construction, the PCR mixture system (50 *μ*L) contained 30 ng of DNA template, 4 *μ*L of the PCR primer cocktail, 25 *μ*L of PCR master mix (NEB Phusion High-Fidelity PCR Master Mix), and an appropriate volume of ddH2O. Amplification of each sample was performed in triplicate. The amplicons were analyzed using 2% agarose gels, purified with the AxyPrep DNA Gel Extraction Kit (Axygen Biosciences, Union City, CA, USA), and quantified using QuantiFluor-ST (Promega, Madison, WI, USA) according to the manufacturer's instructions, and sequencing was then performed with an Illumina HiSeq platform (Illumina, San Diego, CA, USA). The sequencing data were filtered, trimmed, and used for the clustering of operational taxonomic units (OTUs) and taxonomic analysis. At the 97% similarity level, the final OTUs were generated based on the clustering results using Usearch (version 7.1). Weighted UniFrac distance-based PCoA was performed using the R package.

RETRACTED

### 2.8. cAMP Signaling Pathway Verification

The proteins in the total cell lysate were separated using 12% sodium dodecyl sulfate-polyacrylamide gel electrophoresis (SDS-PAGE) and were then transferred onto a polyvinylidene fluoride (PVDF) membrane. The membranes were blocked with 5% skim milk at 37°C for 2 h, washed with Tris-buffered saline and Tween 20 (TBST) buffer, and then probed with primary antibodies overnight at 4°C using *β*-actin as a loading control. After incubation with the appropriate secondary antibodies for 1 h at 37°C, protein bands were visualized using a chemiluminescence imaging system for quantitative analysis.

### 2.9. Statistical Analysis

Results are presented as the mean ± SEM. The statistical significance was analyzed using the GraphPad Prism 6.02 software (GraphPad Software Inc., San Diego, CA, USA). Statistical comparisons of western blot and MWM data were analyzed by two-tailed Student's *t*-test using the Statistical Package for Social Science program (SPSS 22.0, Chicago, IL, USA), and *p* < 0.05 was considered statistically significant.

## 3. Results

### 3.1. Main Compounds of DST

The main compounds of DST were identified by LC-MS. Under the present chromatographic and MS conditions, the compounds showed good separation within 30 min (Figure 1). The mass, retention time, and intensity of the peaks in each chromatogram were detected by TF. Only the compounds whose peak areas showed a higher signal than an established threshold (5.0 × 106) were considered the main compounds of DST. Comparisons with accurate mass and MS/MS data of natural products in OTCML databases identified a total of 80 main compounds in DST; however, some of the compounds were isomers, and thus, the retention time of the reference substance was used to distinguish the isomers. The 10 ginsenosides with isomers were identified by matching with the reference substance, marked on the spectrum, and were found at a high level in DST. The details of the main compounds identified in this study are summarized in Table 1.

### 3.2. Effect of DST on Rats in the Morris Water Maze Test

In the MWM, animals use their survival instinct to find an escape platform, and this test can thus be used to evaluate the spatial memory and learning abilities of rats. The trajectories of the rats in the model group were more complicated than those of the rats in the control group, and after DST treatment, the trajectories of the treated rats approached those of the rats in the control group (Figures 2(a)–2(c)). The time that the rats in the model group needed to find the platform was significantly higher than that of the rats in the control group (*p* < 0.01), and that of the rats in the DST group was significantly shorter than that of the rats in the model group (*p* < 0.01) (Figure 2(d)). These findings suggest that DST could improve the spatial learning, memory, and cognitive abilities of rats with D-gal-induced memory impairment.

RETRACTED

### 3.3. Effects of DST Treatment on the Ultrastructure of the Rat Hippocampus

To evaluate the protective effect of DST, the ultrastructure of neurons in the hippocampus of D-gal-induced rats was assessed by TEM. As shown in Figures 3(a) and 3(d), the hippocampal neurons of the rats in the control group were complete, clear, and well defined. These neurons exhibited a regular nuclear morphology, a smooth nuclear membrane, evenly distributed chromatin, clear nucleoli, abundant organelles, and normal-sized mitochondria. The model group showed obvious neuronal edema in the hippocampus; specifically, the perinuclear body was vacuolated, the nuclear envelope was ruptured, the electron density was high, the area of edema was enlarged, and mitochondria and other organelles were swollen (Figures 3(b) and 3(e)). Compared with those of the model rats, the hippocampal neurons of the rats in the DST group had a complete nuclear membrane, a uniform chromatin distribution, and normal-sized and normal-shaped mitochondria and organelles, which suggests that DST could reduce the neuronal damage in the hippocampus of rats with memory impairment (Figures 3(c) and 3(f)).

### 3.4. Metabolomic Profiling

It is important to verify the reproducibility and stability of the LC-MS method in metabolomic analysis [25]. Therefore, each QC sample was analyzed every six analytical runs to obtain a dataset for assessment of the reproducibility and stability of the method. Furthermore, after obtaining all the peaks from the serum samples and their alignment and normalization, the dataset containing information on the peaks of all the samples was used for PCA. As shown in Figure 4, the QC samples were clustered relatively tightly in comparison with all the samples, and this finding was obtained in both the positive and negative ion modes, which shows the reproducibility and stability of the LC-MS method.

RETRACTED

The serum samples were analyzed by UPLC-Q-TOF/MS, and the raw data were subjected to multivariate statistical analysis through SIMCA-P to reveal the metabolite changes among the three groups and to evaluate the protective effect of DST against memory impairment. The differences in the metabolic profiles among the control, model, and DST groups were visualized by partial least squares-discriminant analysis (PLS-DA), and the results of the permutation test (*n* = 100) shown in Figure S1 revealed that the value of intercepts to the left was lower than the original value, which suggests that the established model was not overfit. The PLS-DA score plots (Figures 5(a) and 5(b)) showed that the model and control groups were completely separated by the principal components in both the positive and negative ion modes, which suggests that the blood metabolism of rats was disordered after model establishment. Furthermore, the cluster of the DST group was located far from that of the model group (Figures 5(c) and 5(d)), which indicates the protective effect of DST on memory repair, and this finding was consistent with the TEM and MWM findings.

The fold change (FC), *p* values, and VIP values were used to select metabolites with the greatest contribution to the separation between the control and model groups. A total of 33 metabolites, with *p* < 0.05 and FC > 2 or FC < 0.5, were identified as candidate biomarkers in the positive and negative ion modes. The structures of these candidate biomarkers were tentatively assigned by comparing the MS and MS/MS spectra with the detected metabolites in the Human Metabolome Database (HMDB), and the detailed information is shown in Table S1. Most of these candidate biomarkers were related to oxidative stress, neuroprotection, mitochondrial disorders, and A*β* deposition, which are involved in the pathogenesis of AD, and most of the metabolic pathways involving these candidate biomarkers were related to the body's energy supply (Table S2). The candidate biomarkers with a VIP value larger than 1 were regarded as potential biomarkers (Table 2).

A heatmap was used to visualize the changes in the potential biomarkers among the groups and the clustering of the potential biomarkers (Figure 6). The color differences between the control and model groups indicate metabolic perturbations in the blood of rats with memory impairment, whereas in the rats treated with DST, the levels of these metabolites were partially recovered to those in the control group.

To reveal the metabolic pathways affected by memory impairment, a pathway analysis of the potential biomarkers was performed through a search of the KEGG database, and the results were visualized using R. The results showed that the relevant pathways influencing memory impairment, including pyruvate metabolism, synthesis and degradation of ketone bodies, pantothenate and CoA biosynthesis, glutathione metabolism, beta-alanine metabolism, butanoate metabolism, and histidine metabolism, were the most important metabolic pathways (Figure 7). By using Impala tools to analyze the signaling pathways involved in potential biomarkers, we found that 3-hydroxybutyric acid and lactic acid were involved in the activation of cAMP signaling pathways.

RETRACTED

### 3.5. Microbial Community Analysis

After the blood metabolomics study, we also studied the effect of DST on the gut microbiota of D-gal-induced rats by performing 16S gene sequencing and found that the alterations induced by DST in the intestinal flora were mainly reflected at the genus level. The clustering of the microbiota structure in the different groups by weighted UniFrac distance-based PCoA showed good separation. The microbial composition of the rats with D-gal-induced memory impairment showed different clusters than that of the rats in the model group (Figure 8(a)). Furthermore, the abundance of microorganisms showed partial variation between the control and model groups, and DST treatment exerted a corrective effect on the abundances of some microbes, such as *Lactobacillus* and *Bacteroides* (Figure 8(b)). In addition, changes in the main microbial structure composition were found among the three groups (Figure 8(c)). In detail, *Ruminiclostridium*, *Butyrivibrio*, *Cyanobacteria_f_norank*, *Cyanobacteria_o_norank*, and *Cyanobacteria_g_norank* were the main functional microorganisms in the control group, and *Porphyromonadaceae*, *Anaerofilum*, *Corynebacterium_1*, *Flavonifractor*, *and Corynebacteriaceae* were the main functional microorganisms that showed alterations in the model group compared with the control group. Importantly, *Peptostreptococcaceae*, *Romboutsia*, *Clostridium_sensu_stricto_1*, *Clostridiaceae_1*, and *Hydrogenoanaerobacterium* were the main functional microorganisms identified in the DST group.

KEGG functional prediction analysis was performed using 18 different microbes at the genus level. The annotated pathways represented potential pathways associated with the changes in the intestinal microbiota observed in the presence of memory impairment (Figure 9). These differential microbes were mainly related to energy metabolism, drug metabolism, other enzymes, signal transduction mechanisms, and sulfur relay systems.

### 3.6. The Influence of DST on Key Proteins in the cAMP Signaling Pathway

Our metabolomics study showed that the DST regulates energy-related especially cAMP signaling pathway. In order to validate the effect of DST on the cAMP signaling pathway, we evaluated additionally the expression of related proteins. As shown in Figure 10, the expression levels of cAMP, PKA, and ADCY, which are closely related to the nerve regeneration, were significantly reduced in the brain tissue of the rats in the model group compared with that in the control group (*p* < 0.05). Meanwhile, the expression level of GNAI was significantly increased in the brain tissue of the model group rats (*p* < 0.05). After DST treatment, the expression levels of cAMP, PKA, and ADCY were significantly increased (*p* < 0.05), while the expression level of GNAI was significantly reduced (*p* < 0.05). These results suggest that the DST improved memory impairment of the aging rats by activating the cAMP signaling pathway. Additionally, the expression of CREB and BDNF was detected, which two proteins are related to the cognitive function and are the downstream target of PKA. The results showed that compared with that in the control group, the expression of CREB and BDNF as significantly reduced in the brain tissue of the model group rats. After DST treatment, the expression of CREB and BDNF was significantly increased, indicating that DST can improve cognitive function and protect neurons by activating cAMP/PKA/CREB signaling pathways.

RETRACTED

## 4. Discussion

Aging leads to brain damage and affects the quality of life of elderly populations, and DST is a widely used herbal decoction for senile diseases in China. In this study, the chemical profiles of DST were investigated by LC-MS-based chemical profiling. A total of 80 major ginsenosides were unambiguously identified in the DST group, and these included ginsenosides R1, Rg1, and Re. The MWM test and TEM analysis were used to assess the potential therapeutic effect of DST against memory impairment, and the results suggested that DST exerted good protective effects against D-galactose-induced memory impairment in rats. Subsequently, serum and fecal samples were analyzed by UPLC-MS and 16S rDNA sequencing to explore the mechanism through which DST affects metabolism and the intestinal flora to protect against cognitive impairment. Consistent with the MWM and TEM results, the PLS-DA score plot of the metabolites and PCoA score plot of the gut microbiota showed that the cluster of the DST group was separated from that of the model group. The metabolic results indicate that many endogenous energy-related metabolites (such as lactic acid and 3-hydroxybutyrate) that were dysregulated in the D-gal-induced rats could be corrected by the DST. The KEGG metabolic pathway analysis indicated that DST mainly regulates pyruvate metabolism and the synthesis and degradation of ketone bodies in rats with memory impairment. It was found that 3-hydroxybutyric acid and lactic acid were involved in the activation of cAMP signaling pathways.

RETRACTED

Our study found that the levels of lactic acid, as an important biomarker of memory impairment, were increased in rats with memory impairment induced by D-gal. Lactic acid, which is the terminal product of lactic acid fermentation, is bioenergetically inefficient but favored under anoxic/hypoxic conditions and in pathological metabolic states [26]. Previous studies have confirmed that lactic acid is not only an energy substrate used preferentially by neurons but also plays an important role in memory formation [27], and this compound is found at higher levels in the frontal cortex and caudate nucleus of patients with AD [28]. These results are consistent with our findings.

It has been confirmed that patients with AD present with mitochondrial dysfunction and metabolic changes [29]. Mitochondrial dysfunction and a decline in respiratory chain function alter amyloid precursor protein processing, which leads to the production of pathogenic amyloid-*β* fragments [30–32]. Mitochondrial disorders are one of the main pathogenic factors of AD, and the size and shape of the mitochondria and organelles return to normal after DST treatment, which suggests the protective effect of DST [33, 34]. Lactic acid accumulation was observed in the model group with memory impairment, and this accumulation might have been observed due to decreased pyruvate dehydrogenase activity, which results in decreased catabolism of lactic acid and reduced mitochondrial respiration and thereby mitochondrial failure. Mitochondrial failure results in intracellular pH changes, synaptic dysfunction, amyloid deposition, and ultimately apoptosis [35, 36].

Mitochondrial dysfunction during aging is a trigger that induces many age-related changes in energy metabolism. Lactate and pyruvate are key intermediates in intracellular energy metabolic pathways and can indicate age-related imbalances in energy metabolism [37]. Lactate prevents cell aging through its lactate dehydrogenase-catalyzed oxidation to pyruvate, and pyruvate inhibits cell aging via its intramitochondrial metabolism [38]. This research has shown that DST can improve memory impairment in aging rats by regulating the metabolism of pyruvate. The mechanism of action of DST might involve acceleration of the oxidation of pyruvate by lactic acid to produce nicotinamide adenine dinucleotide (NADH) and inhibit cell senescence. NADH is then converted into ATP through mitochondrial electron transfer and thereby provides energy to the cell [39]. Ketone bodies commonly refer to 3-hydroxybutyric acid together with acetoacetate and acetone [40] and exert neuroprotective effects on aging brain cells [30]; thus, CoA biosynthesis is highly correlated with energy metabolism. Notably, 3-hydroxybutanoic acid exerts a neuroprotective effect that supports the mitochondrial respiration system by reversing the inhibition of mitochondrial complex I or II [41]. High levels of 3-hydroxybutanoic acid have been shown to improve cognitive function in elderly and memory-impaired subjects [42, 43]. Additionally, 3-hydroxybutanoic acid can replace glucose as the major central nervous system fuel for the brain in humans [44], decrease oxidative stress by binding to specific receptors [45], promote the expression of brain-derived neurotrophic factor [46], and increase cerebral blood flow [47]. In our study, we found that DST increased the serum level of 3-hydroxybutyric acid, which confirmed that DST exerts beneficial effects on memory impairment by regulating the expression of 3-hydroxybutanoic acid and the related energy metabolism.

RETRACTED

Additionally, according to our 16S rDNA sequencing results, we found that DST could correct the disturbance of the gut microbiota, including *Lactobacillus*, *Bacteroidales*, and *Bacteroides*, to improve the memory impairment induced by D-gal (Figure 8(b)). According to published references, *Bacteroidetes* are typically beneficial to human health due to their multiple capabilities, such as supporting glucose homeostasis [48–50], biosynthesizing polysaccharides, and transporting proteins, volatile fatty acids, and other nutrients [51, 52]. *Lactobacillus* can increase the activity of glutamate-cysteine ligase and the rate of glutathione synthesis, block superoxide anion and hydroxyl radical production, decrease the prooxidant content, and stimulate and reinforce the immune system [53–55]. In addition, by improving oxidative stress and neuroinflammation, *Lactobacillus* and *Bacteroidales* can clear plaques and decrease the plaque size and number [56]. *Lactobacillus* is mainly composed of probiotics, which can adjust the composition of the gut microflora and affect the gut barrier function [57]. *Lactobacillus* also leads to lower oxidative stress and inflammatory markers, both of which are the main factors responsible for aging, by affecting cytokine production [58–60]. *Lactobacillus* strains could exert the same mimetic antiaging effects of calorie restriction without an actual reduction in the calorie intake. AMPK can also be regarded as a novel AMPK activator [61] and regulates the dynamics of mitochondria to overcome oxidative stress by minimizing energy consumption and the exhaustion of resources, which results in the restoration of metabolic functions [62]. Furthermore, consistent with the metabolomics findings, the KEGG functional prediction analysis of the intestinal microbiota suggested that the important species of the gut microbiota that were regulated by DST (such as *Lactobacillus* and *Bacteroides*) are also mainly related to oxidative stress and energy metabolism, such as pyruvate, and the synthesis and degradation of ketone bodies.

RETRACTED

Our study validated the effect of DST on cAMP signaling pathways from the protein expression. The cAMP is an important second messenger that mainly activates downstream cAMP-dependent protein kinase A (PKA) and promotes further activation of transcription factors, by which way fundamentally involves in brain mechanisms that require for the neuronal activity, nerve regeneration, energy production, metabolic processes, and synaptic physiology [63, 64]. In the cAMP signaling pathway, the transformation from ATP into cAMP is regulated by the ADCY, and the GNAI as the upstream target of ADCY prevents the generation of cAMP by inhibiting ADCY. The insufficient expression of ADCY by the D-gal induction can lead the reduction of the cAMP expression. The attenuated expression of the cAMP may further lead to the protein kinase (PKA) inactivation, following which to inhibit the expression of phosphorylated cAMP response element binding protein (CREB) [65]. The CREB is a molecular switch that is the core component of long-term memory. The reduction of CREB leads to a decline in memory ability. The phosphorylated CREB can stimulate the expression of brain-derived neurotrophic factor (BDNF), which belongs to neurotrophin family and is involved in learning and memory [66]. Our study found that the DST treatment promoted brain repair by participating protein synthesis for activating cAMP signaling pathway, especially by inhibiting the GNAI to activate the ADCY, following which to further activate its downstream target of cAMP and PKA, as well as the CREB and BDNF in rat brain tissue [67].

## 5. Conclusions

In conclusion, DST significantly improved the spatial memory and learning abilities of model rats and reduced the neuronal damage in the hippocampus of rats with memory impairment induced by D-gal. The 10 potential biomarkers identified by metabolomic analysis were related to pyruvate metabolism, the synthesis, and degradation of ketone bodies, pantothenate and CoA biosynthesis, and other metabolic pathways and were thus mainly related to energy metabolism. These biomarkers also play multiple functions in regulating oxidative stress, neuroprotection, mitochondrial disorders, and A*β* deposition related to aging and AD diseases. Furthermore, 16S rDNA sequencing followed by KEGG functional prediction analysis confirmed that the important species of the gut microbiota influenced by DST (such as Lactobacillus and Bacteroides) are also mainly related to oxidative stress and energy metabolism. In addition, this study has shown that DST inhibits nerve damage and exerts its antiaging effects by activating the cAMP signaling pathway.

RETRACTED

## Figures and Tables

**Figure 1:** TIC chromatograms of Dushen Tang (DST).

**Figure 2:** Effects of Dushen Tang (DST) on the escape latency and path traces in the Morris water maze test. (a–c) Path traces of each group in the Morris water maze test: (a) control group, (b) model group, and (c) Dushen Tang (DST) group. (d) Latency (time) in the Morris water maze test. All the values are expressed as the means (±SDs); ^##^*p* < 0.01 vs. the control group; ^∗∗^*p* < 0.01 vs. the model group.

**Figure 3:** Ultrastructure of hippocampal neurons visualized under a transmission electron microscope. (a–c) Images at 1000x magnification, scale bar = 5.0 *μ*m. (d–f) Images at 3000x magnification, scale bar = 1.0 *μ*m.

**Figure 4:** Principal component analysis (PCA) score plot of all the samples (○) highlighting the quality control (QC) (■) samples in the (a) positive and (b) negative ion modes.

**Figure 5:** Partial least squares-discriminant analysis (PLS-DA) score plots of the control group (▲), model group (red hexagon), and Dushen Tang (DST) group (black diamond) based on data acquired in the (a, c) positive ion mode and in the (b, d) negative ion mode.

**Figure 6:** Heatmap showing the changes in the intensities of potential biomarkers.

**Figure 7:** Bubble plots showing the altered metabolic pathways in rats with memory impairment.

**Figure 8:** Fecal microbiota structure of the different groups. (a) Principal coordinates analysis (PCoA) plots of operational taxonomy units (OTUs) among the control group, model group, and Dushen Tang (DST) group. (b) Bacterial taxonomic profiling of the gut microbiota at the genus level in the different groups. (c) Differentially abundant microbial cladogram obtained by linear discriminant analysis effect size (LEfSe).

**Figure 9:** KEGG functional prediction analysis of the intestinal microbiota. The data are expressed as the means ± SEMs. The analysis shows the relative abundance of microbial genera based on Welch's test (*p* < 0.05). The colored circles represent 95% confidence intervals calculated using Welch's inverted method.

**Figure 10:** Expression levels of cAMP signal pathway-related proteins in rat brain tissues. The data are expressed as the means ± SEMs; ^#^*p* < 0.05 vs. the control group; ^∗^*p* < 0.05 vs. the model group.

RETRACTED

**Table 1:** Details of the compounds identified from DST.

No.	Target name	RT (min)	Formula	Expected (m/z)	Measured (m/z)	Peak number
1	Ginsenoside R1	8.18	C47H80O18	977.5327	977.531	1
2	Ginsenoside Rg1	8.47	C42H72O14	845.4904	845.4893	2
3	Ginsenoside Re	8.53	C48H82O18	991.5483	991.5465	3
4	Ginsenoside Rf	11.28	C42H72O14	845.4904	845.4893	4
5	Ginsenoside Rh1	12.78	C36H62O9	683.4376	683.4371	5
6	Ginsenoside Rb1	14.42	C54H92O23	1153.6011	1153.5995	6
7	Ginsenoside Rc	15.72	C53H90O22	1123.5906	1123.5895	7
8	Ginsenoside Ro	16.08	C48H76O19	955.4908	955.4901	8
9	Ginsenoside Rb2	16.94	C53H90O22	1123.5906	1123.5895	9
10	Ginsenoside Rb3	17.43	C53H90O22	1123.5906	1123.5895	10
11	Ginsenoside Rg2	26.62	C42H72O13	829.4955	829.4958	-
12	Mogroside II A2	11.33	C42H72O14	835.4616	835.4617	-
13	Notoginsenoside Fe	26.24	C47H80O17	961.5378	961.5386	-
14	Tenacissoside H	26.57	C42H66O14	793.438	793.4388	-
15	Cornuside	11.41	C24H30O14	577.133	577.135	-
16	Procyanidin B1	11.41	C30H26O12	577.1351	577.135	-
17	Tomatine	9.25	C50H83NO21	1032.5385	1032.5455	-
18	Picroside II	10.57	C23H28O13	547.1224	547.1248	-
19	Atractyloside A	8.62	C21H36O10	493.229	493.229	-
20	Dehydroandrographolide	26.86	C20H28O4	377.197	377.2005	-
21	Periplocin	12.14	C36H56O13	731.3415	731.3425	-
22	Melittoside	1.01	C21H32O15	523.1668	523.1701	-
23	Araloside A	17.65	C47H74O18	925.4802	925.481	-
24	Tubeimoside I	12.81	C63H98O29	1377.6332	1377.6445	-
25	Geniposidic acid	0.67	C16H22O10	373.114	373.1176	-
26	20(S)-Ginsenoside Rh2	28.76	C36H62O8	621.4372	621.4373	-
27	Orcinol gentiobioside	1.71	C19H28O12	447.1508	447.1512	-
28	Artemisinic acid	27.00	C15H22O2	233.1547	233.1543	-
29	Anemoside B4	14.66	C59H96O26	1219.6117	1219.6201	-
30	Demethylwedelolactone	26.77	C15H8O7	334.9964	334.9937	-
31	Dioscin	8.47	C45H72O16	913.4802	913.4755	-
32	Morroniside	1.44	C17H26O11	451.1457	451.1464	-
33	Licochalcone A	0.67	C21H22O4	373.1212	373.1176	-
34	Gracillin	12.02	C45H72O17	883.4697	883.4666	-
35	Tacrolimus	28.76	C44H69NO12	848.4802	848.4834	-
36	Eupalinolide A	1.01	C24H30O9	461.1817	461.1802	-
37	Jujuboside A	16.94	C58H94O26	1205.5961	1205.5946	-
38	Hosenkoside K	9.16	C54H92O25	1139.5855	1139.585	-
39	Methyl hexadecanoate	26.89	C17H34O2	315.2541	315.2543	-
40	Polyphyllin E	8.53	C51H82O20	1059.5382	1059.5337	-
41	Dihydrocucurbitacin F	27.03	C30H48O7	565.3382	565.3344	-
42	Asiaticoside	16.23	C48H78O19	957.5064	957.4971	-
43	Periplocymarin	18.35	C30H46O8	569.2887	569.2898	-
44	Macranthoside B	26.33	C53H86O22	1073.5538	1073.5568	-
45	Momordin Ic	26.74	C41H64O13	763.4274	763.4285	-
46	Kanzonol C	11.26	C25H28O4	391.1915	391.1888	-
47	Doxorubicin hydrochloride	11.41	C27H30NO11Cl	578.1435	578.1383	-
48	Morin	26.71	C15H10O7	337.012	337.0092	-
49	Obacunone	6.57	C26H30O7	499.1974	499.1954	-
50	Forsythoside E	3.59	C20H30O12	461.1664	461.1671	-
51	Ginsenoside Rk1	27.00	C42H70O12	765.4794	765.4786	-
52	Raddeanin A	9.23	C47H76O16	931.4827	931.4911	-
53	Protodioscin	8.82	C51H84O22	1047.5382	1047.5389	-
54	Sibiricose A6	2.06	C23H32O15	547.1668	547.1677	-
55	Ginsenoside Rh2	26.97	C36H62O8	667.4427	667.4435	-
56	Madecassoside	9.72	C48H78O20	973.5014	973.4927	-
57	Qingyangshengenin	7.90	C28H36O8	535.2104	535.2148	-
58	Arctiin	7.32	C27H34O11	579.2083	579.208	-
59	Cucurbitacin B	15.48	C32H46O8	593.2887	593.2876	-
60	L-Tryptophan	0.86	C11H12N2O2	203.0826	203.082	-
61	Ophiopogonin D	7.45	C44H70O16	853.4591	853.4564	-
62	Polyphyllin I	7.45	C44H70O16	853.4591	853.4564	-
63	Artesunate	1.89	C19H28O8	419.1478	419.1501	-
64	Morusin	1.89	C25H24O6	419.15	419.1501	-
65	Loganin	0.95	C17H26O10	389.1453	389.146	-
66	Handelin	9.02	C32H40O8	597.2705	597.2689	-
67	Gypenoside A	26.62	C46H74O17	897.4853	897.4833	-
68	Sophoricoside	7.21	C21H20O10	477.1038	477.1042	-
69	Eleutheroside B/syringin	1.01	C17H24O9	417.1402	417.1404	-
70	Gomisin D	6.27	C28H34O10	529.2079	529.2064	-
71	Helicid	0.50	C13H16O7	329.0878	329.0879	-
72	Iso-astragaloside I	11.28	C45H72O16	903.4514	903.4485	-
73	11-Oxomogroside V	13.76	C60H100O29	1283.6278	1283.6276	-
74	6-Shogaol	27.00	C17H24O3	275.1653	275.1654	-
75	Pseudoprotodioscin	8.05	C51H82O21	1075.5331	1075.5281	-
76	Vincristine sulfate	12.01	C46H56N4O10	869.3978	869.4009	-
77	Digitonin	16.11	C56H92O29	1263.5418	1263.5448	-
78	Irinotecan hydrochloride	8.05	C33H39N4O6Cl	585.2719	585.2675	-
79	Engeletin	7.19	C21H22O10	433.114	433.1142	-
80	Lanatoside C	8.21	C49H76O20	1029.4912	1029.4956	-

RETRACTED

**Table 2:** Annotated potential biomarkers and the trends of their changes in serum.

No.	Compound name	m/z	Formula	Adduct	VIP	Model/control	DST/model
1	8-Hydroxycarapinic acid	509.15598	C26H30O8	[M+H]+	1.05956	↓^∗^	↑^###^
2	Pantothenic acid	220.11649	C9H17NO5	[M+H]+	1.93711	↓^∗^	↑
3	Creatinine	114.06604	C4H7N3O	[M+H]+	3.9793	↑^∗^	↓
4	Erucamide	338.33859	C22H43NO	[M+H]+	5.24912	↑^∗∗∗^	↓^##^
5	Threonic acid	135.02975	C4H8O5	[M-H]-	1.07714	↓^∗^	↑
6	Anserine	239.11552	C10H16N4O3	[M-H]-	3.35603	↓^∗^	↑^#^
7	3-Hydroxybutanoic acid	103.03831	C4H8O3	[M-H]-	4.24771	↓^∗^	↑
8	Phenacylamine hydrochloride	170.04254	C8H10ClNO	[M-H]-	2.82537	↓^∗^	↑^#^
9	Chlorothalonil-4-hydroxy	244.90831	C8HCl3N2O	[M-H]-	2.04014	↓^∗∗^	↑^#^
10	DL-Lactic acid	89.02377	C3H6O3	[M-H]-	3.35603	↑^∗^	↓

^∗^ *p* < 0.05, ^∗∗^*p* < 0.01, and ^∗∗∗^*p* < 0.001, the model group versus the control group; ^#^*p* < 0.05, ^##^*p* < 0.01, and ^###^*p* < 0.001, the Dushen Tang (DST) group versus the model group.

## Data Availability

All data are provided in this study, and raw data can be requested to the corresponding author.

## Supplementary Materials

Supplementary Materials Figure S1: PLS-DA of the control and model groups based on the data obtained in the (a) positive ion mode and (b) the negative ion mode; PLS-DA of the model and DST groups based on the data obtained in the (c) positive ion mode and (d) the negative ion mode. Table S1: candidate biomarkers and their mode of action that might be related to memory impairment. Table S2: list of metabolic pathways related to candidate biomarkers (*p* < 0.05).
